# Parecoxib inhibits esophageal squamous cell carcinoma progression via the PDK1–AKT pathway

This article has been retracted.

**DOI:** 10.1186/s11658-022-00324-w

**Published:** 2022-03-19

**Authors:** Han-Ming Huang, Xiao-Yu Huang, Shao-Ping Wu, Can-Keng Chen, Xin-Hua He, Yong-Fa Zhang

**Affiliations:** 1 Department of Anesthesiology, Second Affiliated Hospital of Shantou University Medical College, Shantou, 515041 People’s Republic of China; 2 Department of Physiology, Shantou University Medical College, Shantou, 515041 People’s Republic of China

**Keywords:** Parecoxib, Mutant p53, PDK1–AKT, ESCC

## Abstract

**Background:**

Parecoxib plays an important role in inhibition of human cancer. However, the effect of parecoxib on esophageal squamous cell carcinoma (ESCC) is still not well known. The purpose of this study was to investigate the effect of parecoxib on ESCC and its underlying mechanism.

**Methods:**

RNA-sequence analysis was performed to identify functional alterations and mechanisms. Cell cycle, proliferation, invasion, and migration were assessed using flow cytometry, CCK-8 assay, colony formation, transwell, and wound healing assays. Extracellular matrix (ECM) degradation was detected by substrate gel zymography and 3D cell culture assay. Western blotting was used to detect parecoxib-dependent mechanisms involving cell cycle, proliferation, invasion, and migration. Tumor formation in vivo was detected by mouse assay.

**Results:**

Functional experiments indicated that parecoxib induced ESCC cell cycle arrest in G2 phase, and inhibited cell proliferation, invasion, and migration in vitro. Western blotting revealed that parecoxib downregulated the phosphorylation levels of AKT and PDK1, as well as the expression of the mutant p53, cyclin B1, and CDK1, while upregulating p21waf1. Parecoxib inhibited matrix metalloproteinase-2 (MMP2) secretion and invadopodia formation, which were related to ECM degradation. Furthermore, we found that parecoxib suppressed ESCC growth in heterotopic tumor models.

**Conclusion:**

Parecoxib inhibits ESCC progression, including cell cycle, proliferation, invasion, and migration, via the PDK1–AKT signaling pathway.

**Supplementary Information:**

The online version contains supplementary material available at 10.1186/s11658-022-00324-w.

## Background

ESCC accounts for about 90% of the annual 456,000 cases of esophageal cancer worldwide [1]. ESCC is usually diagnosed at an advanced stage, leading to poor prognosis and high mortality. At present, there are no good screening and prevention methods for ESCC [2]. Although treatments for ESCC have improved greatly over the past half-century, long-term survival rate remains grim [3]. For this reason, we hope to find new targets for chemotherapeutic strategies of ESCC.

Cyclooxygenase (COX) is the key enzyme in the conversion of arachidonic acid to prostaglandin, which has two isozymes, namely cyclooxygenase-1 (COX-1) and cyclooxygenase-2 (COX-2) [4]. COX-2 is found in inflammatory, immune, neuronal, and cancer cells [5], and plays a key role in a variety of physiological and pathological processes, including inflammation, neurodegenerative diseases, and cancer progression [6]. COX-2 is a focus of intense research for cancer treatment and is overexpressed in various cancers, including ESCC [6]. COX-2 has been considered as a marker for cancer development.

The antiinflammatory and analgesic effects of nonsteroidal antiinflammatory drugs (NSAIDs) are mainly due to the inhibition of COX activity. Further studies have confirmed that the antiinflammatory and analgesic effects of traditional NSAIDs are the mainly results of COX-2 inhibition [7]. The further clinical development of selective COX-2 inhibitors is due to the fact that the COX-1 inhibition induced by traditional NSAIDs increases the risk of gastrointestinal bleeding [8]. Thus, selective COX-2 inhibitors have been widely used in perioperative analgesia as relatively safe and effective drugs [9]. Simultaneously, some researchers have reported that selective COX-2 inhibitors could reduce recurrence and metastasis in tumor patients after radical surgery. Therefore, selective COX-2 inhibitors have shown anticancer properties in addition to the analgesic effect.

Parecoxib is the most commonly used selective COX-2 inhibitor in the clinic, and is the only parenterally administered coxib available to date [10, 11]. It has been reported that parecoxib could improve the postoperative analgesic effect and immune function when used for multimodal analgesia, and further postpone postoperative cancer recurrence [12, 13]. Other studies have reported that parecoxib shows antitumor effects against human osteosarcoma, glioblastoma, and intestinal cancers [14–16]. Studies have further revealed the important role of parecoxib in the inhibition of vascular formation in cancer. Parecoxib reduces the expression of vascular endothelial growth factor in the tumor microenvironment, which is expected to become a novel strategy for cancer treatment [17].

Epidemiological evidence indicates that prolonged administration of nonselective COX inhibitors can effectively reduce the risk of ESCC [18]. However, application of selective COX-2 inhibitors in chemotherapy for ESCC is rarely reported, and the underlying mechanism is not understood. Therefore, we designed a series of experiments to investigate whether parecoxib could inhibit ESCC progression and aimed to elucidate the possible underlying mechanism.

## Materials and methods

### Cell lines and parecoxib treatments

Human primary ESCC cell lines (KYSE30, 150, 180, and 410) were cultured at 37 °C in a humidified atmosphere of 5% CO_2_ in RPMI 1640 medium (HyClone, USA) containing 10% fetal bovine serum. All cell lines were provided by Professor Li-Yan Xu (Institute of Oncologic Pathology, Medical College of Shantou University, Shantou 515041, PR China). ESCC cell lines were established by Dr. Shimada Yutaka (Faculty of Medicine, Kyoto University, Japan) [19]. Before use, the cell lines were confirmed to be pathogen free. Parecoxib (sodium parecoxib, Dynastat) with purity > 95% was purchased from Pfizer (Da Lian, China), and 0.9% saline was used as a vehicle in both in vitro and in vivo experiments. As determined pre-experiment, parecoxib inhibited ESCC cell proliferation in vitro in a dose-dependent manner, with an IC_50_ of 387 and 322 μM for KYSE30 and KYSE180 cells, respectively. The concentration of parecoxib was set as 0, 100, 200, and 300 μM for in vitro experiments.

### Gene Ontology (GO) and Kyoto Encyclopedia of Genes and Genomes (KEGG) enrichment analysis

KYSE30 cells were seeded on two six-well plates; at the same time, medium with or without 300 μM of parecoxib was added. Twenty-four hours later, 1 ml of TRIzol lysate was added into the cell sample plate. After vortex mixing, the cells were placed at room temperature for 5 min for full lysis. Oligo magnetic beads were used to enrich the mRNA, and interruption reagents were added to fragment the mRNA. The synthesized cDNA chain was added to the interrupted mRNA for synthesis of two-stranded cDNA. The linker products were amplified using PCR reaction system. After denaturing the PCR product into a single chain, the cyclization reaction system was prepared to obtain the final library. The single-stranded circular DNA molecule was replicated by rolling ring, and high-density DNA nanochip technology combined with probe anchoring polymerization was used to obtain 50 bp/100 bp/150 bp sequencing read length. The differentially expressed mRNAs were identified for GO and KEGG pathway analyses. For GO analysis, the differentially expressed genes were classified according to biological process, cellular component, and molecular function. For KEGG analysis, the different pathways were ranked by their enrichment scores.

### Cell migration and invasion assays

Migration and invasion assays were performed using transwell chambers. For invasion assays, 1 × 10^5^ cells were resuspended with serum-free medium containing parecoxib (0, 100, 200, and 300 μM) and seeded onto the top Matrigel-coated chamber with 8-μm pores (BD Falcon, USA) (for the migration assay, cells were directly plated on an uncoated chamber). The bottom of the chamber was filled with medium containing 10% fetal bovine serum. After 24 h (migration assays) or 48 h (invasion assays), we removed the top layer cells in chambers, and the chambers were fixed and stained with hematoxylin (Baso, China). The cell numbers were quantified by counting ten random fields under a microscope (200×, Olympus IX73, Japan).

### Wound healing assay

Cells were seeded on six-well plates and grown to confluence, and cultured with serum-free medium overnight. Cells were scratched with a standard 200 μl pipette tip and washed with serum-free medium to remove cell debris. Subsequently, the scratched cells were cultured with 2% fetal bovine serum medium containing parecoxib (0, 100, 200, and 300 μM). Serial photographs were obtained at different timepoints (0, 12, 24 h) using a microscope (200×, Olympus IX73, Japan). The rate of wound healing was calculated by counting the proportion of 24 h healing area to 0 h scratching area.

### CCK-8 assay

A Cell Counting Kit-8 (CCK-8) assay was conducted to assess cell proliferation. Initially, cells were pretreated with parecoxib (0, 100, 200, and 300 μM), and then 5000 cells were seeded per well of 96-well plates at 37 °C for 6–7 h. Afterwards, CCK-8 solution (Dojindo, Mashikimachi, Japan) was added to the cells for further incubation for 1 h. Absorbance at 450 nm was measured at 24 h using a plate microplate reader (Multiskan FC, Thermo). Raw data were normalized against those of the medium blank control.

### Colony formation assays

For colony formation assays, cells were seeded in six-well plates at 2 × 10^3^ cells per well and cultured with medium containing parecoxib (0, 100, 200, and 300 μM) for 2 weeks. Then, cells were washed three times with phosphate-buffered saline (PBS), fixed with methanol/acetic acid (3:1, v/v), and stained with 0.5% crystal violet (Sigma, China). Photography of colonies was performed using a ChemiDoc XRS + Imaging System (Bio-Rad, USA). The number of colonies was counted with Image J software. Cloning rate was calculated by counting the proportion of clone number to inoculation number.

### Flow cytometry

For flow cytometry, cells were pretreated with parecoxib (0, 100, 200, and 300 μM) for 24 h and washed three times with PBS following trypsinization, and then fixed with 75% precooled ethanol at −20 °C for 48 h. The fixed cells were washed twice with 500 μl PBS, then 3 μl of 10 mg/ml RNase (Sigma, USA) was added. Cells were incubated with RNase solution for 30 min and then stained by adding 1.5 μl of 1 mg/ml PI (Sigma, USA) before detection. Histograms of DNA content were generated by flow cytometry (BD FACSAriaII, USA) and then used to analyze cell cycle distribution using FlowJo V10 software.

### Substrate gel zymography

10% SDS-PAGE gels were prefabricated including 1 mg/ml gelatin (Thermo, USA) and used for gelatin substrate enzyme profiles. Cells were cultured with serum-free medium overnight. After discarding the supernatant, cells were cultured with equal-volume serum-free medium containing parecoxib (0, 100, 200, and 300 μM) for 24 h, and then the supernatant was collected and condensed. The equal amounts of proteins were diluted into 2× Tris–Glycine SDS buffer and separated by electrophoresis under nonreducing conditions. Proteins were allowed to regenerate in regeneration buffer (Thermo, USA) for 30 min, then the gel was incubated in development buffer (Thermo, USA) for 30 min and then overnight in the same buffer at 37 °C. After staining with SimplyBlue SafeStain (Thermo, USA), protease activity was shown as clear bands against a blue background. MMP2 was located near the 70 kDa marker band. Photography of the gel was performed using a ChemiDoc XRS + Imaging System (Bio-Rad, USA). The gray values of bands were analyzed by Image J software.

### 3D cell culture

Matrigel basement membrane matrix (Corning, USA) was used for 3D cell culture. KYSE30 or KYSE180 cells were mixed with Matrigel matrix at 8 × 10^5^ cells/100 μl, which were seeded in six-well plates and cultured in 10% fetal bovine serum medium with parecoxib (0, 100, 200, and 300 μM). Cells were incubated at 37 °C, under 5% CO_2_–95% air, and serial photographs were taken at different timepoints (0, 12, 24 h) to observe the formation of invadopodia by microscope (200×, Olympus IX73, Japan).

### Western blotting

Cell lysates were prepared by mixing RIPA lysis buffer (RIPA; Pierce, Rockford, IL) with 1× Halt Protease and Phosphatase Inhibitor Cocktail (78445, EDTA-free, 100×, Thermo, USA). BCA protein assay kit (Pierce Biotechnology, USA) was used for measuring the protein concentration. Equal amounts of protein were diluted in 2× Tris–glycine SDS buffer and separated by electrophoresis under reducing conditions. Then, proteins were transferred onto PVDF membranes (Roche, Switzerland). The membrane was blocked with nonfat milk diluted in TBST for 1 h at room temperature, then incubated with primary antibodies against COX-2 (1:1000, CST no. 12282), GAPDH (1:5000, Thermo no. MA515738), phospho-AKT (S473) (1:1000, CST no. 4060), AKT (1:1000, CST no. 4691), pPDK1 (1:1000, CST no. 3438), PDK1 (1:1000, CST no. 5662), p53 (1:1000, CST no. 2524), CDK1 (1:1000, Abcam no. ab133327), cyclin B1 (1:1000, CST no. 12231), p21waf1 (1:1000, CST no. 2947), and β-actin (1:5000, Thermo no. MA515452) at 4 °C overnight. After washing with TBST three times (5 min once), membranes were then incubated at room temperature for 2 h with enzyme-conjugated secondary antibody goat anti-rabbit IgG (1:5000, Thermo no. A32731) or secondary antibody goat anti-mouse IgG (1:5000, Thermo no. 31430). GAPDH or β-actin was used as an internal reference. Antigen–antibody complexes were detected using SuperSignal West Pico PLUS Chemiluminescent Substrate (Thermo no. 34578). Photography of the band signals was performed using a ChemiDoc XRS + Imaging System (Bio-Rad). The gray values of bands were analyzed by Image J software.

### In vivo tumor growth assay

All animal experiments complied with the policy of Shantou University on the care and use of laboratory animals. Four-week-old male NU/NU nude mice were obtained (Charles River, China) and bred under specific pathogen-free conditions. 1.5 × 10^7^ KYSE30 cells were subcutaneously injected into the right shoulder of the mice (five mice per group). Parecoxib (0.3 mg/kg) [20] was injected into the enterocoelia every 3 days after tumor cell inoculation. Mice were treated with equal volume of normal saline as the untreated control. After 5 weeks, tumor volume was observed. Upon termination of the experiment, mice were euthanized and tumors were excised.

### Statistical analysis

Statistical analyses were performed with SPSS 17.0 and GraphPad Prism 7.0 software. Data represent mean ± standard deviation of three independent trials. A two-sided Student’s *t*-test was used to compare statistical differences. Differences were considered statistically significant at *P* < 0.05 (*), *P* < 0.01 (**), *P* < 0.001 (***), and *P* < 0.0001 (****).

## Results

### Relative expression of COX-2 in ESCC cell lines and the prediction for function or mechanism after treatment with parecoxib by RNA-seq

We examined COX-2 expression level in four ESCC cell lines by western blotting (Fig. 1A). KYSE30 and KYSE180 cells had higher COX-2 protein levels than KYSE150 and KYSE410. We selected KYSE30 and KYSE180 for the subsequent experiments.

**Fig. 1:** Relative expression of COX-2 in ESCC cell lines and prediction for function or mechanism after treatment with parecoxib. **A** Relative expression of COX-2 was measured in four ESCC cell lines by western blotting. **B** GO analysis of differentially expressed mRNA after treatment with parecoxib (300 μM), suggesting variation in cell cycle, proliferation, and cell adhesion. **C** KEGG analysis of pathways enriched for differentially expressed mRNA, indicating variation in cell cycle, ECM, p53, and pathways in cancer

To explore the potential variation of function after treatment with parecoxib, GO analysis was performed to predict the altered biological processes. The top 20 highest and most significant GO terms were determined by calculating the enrichment score (*P* < 0.05) (Fig. 1B). The red-framed GO terms in Fig. 1B had significant differences, including cell cycle, cell adhesion, and cell proliferation, which were demonstrated in subsequent experiments. KEGG database was used to predict the impact of parecoxib on signaling pathways. Twenty pathways with significant differences (*P* < 0.05) based on aberrant gene expression were identified (Fig. 1C). Four significantly pathways are marked in red frame, and were detected in subsequent experiments.

### Parecoxib induced cell cycle arrest at G2 and inhibited proliferation, invasion, and migration of ESCC cells

To investigate the effect of parecoxib on ESCC cells, flow cytometry was performed to determine cell cycle phase distributions of treated cells. The results showed that parecoxib dose-dependently induced G2 phase arrest with increasing the percentage of KYSE30 cells from 12% to 25.5% and KYSE180 cells from 3.93% to 21.8% (Fig. 2A, B). Colony formation and CCK-8 assays suggested that parecoxib led to suppression of cell proliferation in a dose-dependent manner (Fig. 2C, D). Parecoxib dose-dependently inhibited the invasive ability of ESCC cells in Matrigel-coated transwell assays (Fig. 2E), and inhibited the migratory ability of ESCC cells in dose-dependent manner in both transwell and wound healing assays (Fig. 2F, G).

**Fig. 2:** Parecoxib-induced cell cycle arrest at G2 and inhibition of proliferation, invasion, and migration of ESCC cells. **A**, **B** Cell cycle phase distribution (**A**) and relative cell population (**B**) of parecoxib-treated KYSE30 and KYSE180 cells were determined by flow cytometry. **C** KYSE30 and KYSE180 cells treated with parecoxib (0, 100, 200, and 300 μM) were examined for colony formation. **D** Cell viability was determined by CCK8 assay after 24 h treatment with parecoxib (0, 100, 200, and 300 μM). **E** The difference in invasive ability of KYSE30 and KYSE180 cells treated with parecoxib (0, 100, 200, and 300 μM) was assessed by transwell invasion assay. **F**, **G** The difference in migratory ability of KYSE30 and KYSE180 cells treated with parecoxib (0, 100, 200 and 300 μM) was assessed by transwell migration assay (**F**) and wound healing assay (**G**). Images represent three independent experiments. Data are mean ± standard deviation of three independent experiments. *P < 0.05, **P < 0.01, ***P < 0.001, and ****P < 0.0001

### Parecoxib induced variation in mechanism of cell cycle arrest and inhibition of proliferation, invasion, and migration in ESCC

Examining the impact of parecoxib on signaling pathways in ESCC, we found that the pAKT(S473) and pPDK1 phosphorylation level was significantly decreased after treatment with parecoxib in a dose-dependent manner, in the absence of changes in total protein expression of AKT and PDK1 (Fig. 3A). To confirm the cell cycle arrest at G2, we tested for G2/M-associated proteins. Western blotting showed that the expression of cyclin B1 and CDK1 was decreased after treatment with parecoxib in a dose-dependent manner (Fig. 3B). Additionally, mutant p53 was also dose-dependently decreased after treatment with parecoxib, while p21WAF1 was increased (Fig. 3B). Zymography to investigate ECM-degrading enzymatic activity showed that MMP2 activity was dose-dependently reduced after treatment with parecoxib (Fig. 3C). The data, representing mean ± standard deviation of three independent trials, are shown in Additional file 1: Fig. S1. The 3D cell culture assay demonstrated that parecoxib could inhibit invadopodia formation in ESCC cells (Fig. 3D).

**Fig. 3:** Parecoxib-induced variation in mechanism of cell cycle arrest and inhibition of proliferation, invasion, and migration in ESCC cells. **A** Levels of pAKT(S473) and pPDK1 were decreased after treatment with parecoxib, in the absence of changes in total protein expression of PDK1/AKT by western blotting. **B** The variation of critical regulatory proteins for the transition from G2 to M phase was detected by western blotting. Mutant p53, cyclin B1, and CDK1 were decreased, while p21waf1 was increased. **C**, **D** Parecoxib suppressed ECM degradation of ESCC cells by the inhibition of MMP2 secretion (**C**) and invadopodia formation (**D**). Images represented three independent experiments. Data are mean ± standard deviation of three independent experiments. The data are shown in Additional file 1: Fig. S1. *P < 0.05, **P < 0.01, and ***P < 0.001

### Parecoxib suppressed tumorigenicity in vivo

On the basis of the above results, we investigated whether parecoxib could reduce tumorigenicity in vivo. We injected 1.5 × 10^7^ KYSE30 cells into right shoulder blade of nude mice and injected parecoxib (0.3 mg/kg) or normal saline (the blank) into the enterocoelia every 3 days after tumor cell inoculation, and observed tumor growth (Fig. 4A). Five weeks later, we removed the tumors from heterotopic tumor models and measured their size (Fig. 4B). We found that parecoxib suppressed the tumor volume compared with the control, indicating that parecoxib could inhibit ESCC growth in vivo.

**Fig. 4:** Parecoxib suppressed tumorigenicity in vivo. **A** Tumor formation in nude mice after 5 weeks. 1.5 × 10^7^ KYSE30 cells were injected into the right shoulder blade of nude mice. Parecoxib (0.3 mg/kg) or equal volume of normal saline (the blank group) was injected into the enterocoelia every 3 days after tumor cell inoculation. **B** Tumor tissues were resected from nude mice at 5 weeks post-inoculation

## Discussion

Parecoxib has been reported to regulate biological processes, including proliferation, migration, and invasion of tumor cells [14–17]. Considering the relatively high expression of COX-2 in two ESCC cell lines (KYSE30 and KYSE180) (Fig. 1A), we designed and performed functional assays in vitro and in vivo to detect the effect of parecoxib on ESCC. We found that parecoxib efficiently induced ESCC cell cycle arrest at G2, and inhibited cell proliferation, invasion, and migration in vitro (Fig. 2). Additionally, parecoxib could inhibit tumor growth in heterotopic tumor models (Fig. 4). The results of our study suggest that parecoxib exerts an anticancer effect on ESCC.

Mechanistically, activation of the AKT signaling pathway plays a positive role in human malignant tumor processes, including cell cycle, proliferation, metastasis, and invasiveness of cancer cells [21, 22]. PDK1 is a crucial signaling transducer in the AKT signaling pathway [23]. In our study, we found that the phosphorylation levels of PDK1 and AKT were simultaneously decreased, which indicated that the anticancer effects of parecoxib might be achieved through the PDK1–AKT pathway (Fig. 3A).

The complex of CDK1 and cyclin B1 is responsible for promoting G2-to-M transition. The activity of the CDK1–cyclin B1 complex is associated with the expression levels of CDK1 and cyclin B1 [24]. The results of western blotting showed that parecoxib downregulated the expression of CDK1 and cyclin B1, which suggested that parecoxib could induce cell cycle arrest at G2. Simultaneously, we found that p21waf1 was increased in a dose-dependent manner after treatment with parecoxib (Fig. 3B). It has been reported that p21waf1, regulated by p53, inhibits CDK activity indirectly by interfering with the activating phosphorylation of CDK1 so as to induce cell cycle arrest [25]. Our results seem to indicate that parecoxib induces cell cycle arrest at G2 via p53/p21waf1. Interestingly, we found the expression of p53 was decreased in our study (Fig. 3B). The p53 tumor suppressor is influenced by multiple oncogenic signals and thus regulates a variety of cellular processes, including cell cycle arrest, apoptosis, and senescence [26]. The p53 is now generally recognized as a negative transcription factor inhibiting the transition from G2 to M phase [27]. It has been reported that the p53 tumor suppressor gene has a mutation frequency of approximately 50% in most major cancers [28]. There is research reporting that mutant p53 loses original functions and acquires oncogenic properties in ESCC [29]. Therefore, we speculate the p53 has been mutated in the two ESCC cell lines, acquiring the positive regulation for the transition from G2 to M phase. In vitro [30, 31] and in vivo [32, 33] studies have revealed high levels of mutant p53 protein associated with activated AKT, which, together with genetic studies [34], indicates that the AKT pathway can provide positive regulation of mutant p53 levels in an mdm2-independent manner [35]. The results of our study imply that reduction of mutant p53 expression might be caused by the decreased AKT, but specific mechanisms remain to be investigated.

Cancer metastasis is the main cause of cancer-related death, involving invasion into adjacent tissues and distant organ metastasis. Invadopodia are subcellular structures rich in actin, and are associated with extracellular matrix (ECM), thereby affecting cancer invasion and metastasis [36]. Invadopodia protrude into their underlying matrix and bind to ECM-degrading proteinases [36]. Matrix metalloproteinases (MMPs) belong to the family of ECM-degrading proteinases that contain membrane-anchored MMPs (MT1-MMP) and soluble MMPs (MMP2) [37]. MMP2 are secreted by invadopodia and activated by MT1-MMP. Activated MMP2 diffuses into the extracellular space, further mediating degradation of ECM around the invadopodia [38]. In this study, we demonstrated that parecoxib could inhibit MMP2 secretion and the formation of invadopodia (Fig. 3C, D), which would lead to inhibition of ECM degradation so as to inhibit ESCC invasion and migration. Studies also suggest that the AKT pathway can regulate ECM degradation, angiogenesis, and metastasis [39]. Thus, we speculate that parecoxib regulates ECM degradation via the PDK1–AKT pathway, contributing to invasion and migration of ESCC cells. We illustrate how parecoxib exerts its antitumor effects in the graphic abstract (Fig. 5).

**Fig. 5:** Graphic abstract. Parecoxib regulated cell cycle, proliferation, invasion, and migration via the PDK1–AKT signaling pathway. Specifically, parecoxib induced cell cycle arrest at G2 via PDK1/AKT/mutant p53/p21waf1, and inhibited ECM degradation so as to suppress ESCC invasion and migration

## Conclusions

Clinically, how parecoxib affects cancer patients is still unclear, especially in ESCC. In mouse experiments, we found that parecoxib exerted an antitumor effect in vivo (Fig. 4). In future research, we will determine the functional and mechanistic variations in vivo and clarify the clinical effects of parecoxib. At present, we conclude that parecoxib induces cell cycle arrest at G2 phase, and inhibits ESCC cell proliferation, invasion, and migration via the PDK1–AKT signaling pathway, indicating that parecoxib is potentially a novel antitumor and analgesic therapeutic for ESCC patients.

## Supplementary Information

**Additional file 1: Figure S1.** Statistic data of WB and Gel.

## Data Availability

Not applicable.

## Abbreviations

ESCC: Esophageal squamous cell carcinoma
ECM: Extracellular matrix
MMP2: Matrix metalloproteinase-2
MMPs: Matrix metalloproteinases
COX: Cyclooxygenase
COX-1: Cyclooxygenase-1
COX-2: Cyclooxygenase-2
NSAID: Nonsteroidal antiinflammatory drug
GO: Gene Ontology
KEGG: Kyoto Encyclopedia of Genes and Genomes
CCK-8: Cell Counting Kit-8
PBS: Phosphate-buffered saline
